# Finger Vein Verification on Different Datasets Based on Deep Learning with Triplet Loss

**DOI:** 10.1155/2022/4868435

**Published:** 2022-10-20

**Authors:** Jun Li, Luokun Yang, Mingquan Ye, Yang Su, Juntong Liu

**Affiliations:** ^1^School of Medical Information, Wannan Medical College, Wuhu, Anhui 241002, China; ^2^Anhui Provincial Key Laboratory of Network and Information Security, Anhui Normal University, Wuhu, Anhui 241002, China

## Abstract

In this study, deep learning and triplet loss function methods are used for finger vein verification research, and the model is trained and validated between different kinds of datasets including FV-USM, HKPU, and SDUMLA-HMT datasets. This work gives the accuracy and other evaluation indexes of finger vein verification calculated for different training-validation set combinations and gives the corresponding ROC curves and AUC values. The accuracy of the best result has reached 98%, and all the ROC AUC values are above 0.98, indicating that the obtained model can identify the finger veins well. Since the experiments are cross-validated between different kinds of datasets, the model has good adaptability and applicability. From the experimental results, it is also found that the model trained on the dataset that is more difficult to be distinguished will be a better and more robust model.

## 1. Introduction

With the development of economy and the advancement of science and technology, information security has attracted increasing attention, and identity authentication based on biological characteristics is a popular research direction in the field of information security [1]. Common biometrics includes face, fingerprint, voice, iris, palm vein, finger vein, and gait. As an emerging biometric verification technology, finger vein features have the following outstanding advantages [2]. Finger vein features can only be collected when blood is flowing. When a person loses life, blood stops flowing, and finger vein images cannot be collected at this time; finger vein authentication obtains the information of the vein inside the finger, not the information on the surface of the finger, so the wear, humidity, and cleanliness of the finger surface will not cause verification obstacles; the finger vein needs to be collected under infrared light, which is difficult to be stolen, and the veins of the human body are very complicated and difficult to be copied or forged. In general, biometric verification, including finger vein verification, is more secure, confidential, and convenient.

There have been many works related to finger vein feature extraction. Miura et al. proposed a method to extract finger vein patterns using maximum curvature points [3]. Huang et al. introduced a wide line detector method that can obtain the width information of finger veins [4]. Miura et al. also proposed a repeated line tracking method to extract the texture features of finger veins [5]. Choi et al. proposed a principal curvature calculation method that can effectively extract finger vein patterns regardless of vein thickness or brightness [6]. Matsuda et al. proposed a method based on feature point matching to combat changes in finger pose and illumination [7]. Lee et al. used the local binary pattern method to extract finger vein codes and achieved good verification results [8]. Mahri et al. implemented a phase correlation function to match finger vein images [9]. Recently, there have been a lot of related works on finger vein verification using deep learning. Hu et al. gave an FV-net to learn the more discriminative and robust feature representations of finger veins [10]. Hong et al. proposed a method based on the modified VGGNet16 network for finger vein verification and achieved good verification results [11]. Zhang et al. proposed adaptive Gabor convolutional neural networks to decrease the number of parameters of networks for finger vein verification [12].

The traditional finger vein verification methods based on hand-crafted features are more sensitive to image quality and changes in finger posture and illumination and are not very stable. The finger vein verification methods based on convolutional neural network can automatically learn image features from training datasets without hand-crafted design and have a greater improvement in stability and verification accuracy than traditional finger vein verification methods. This work intends to use modified ResNet18 and VGGNet16 networks combined with a triplet loss function to perform finger vein verification and cross-validation on different kinds of datasets. The paper is organized as follows: the next section introduces the datasets and the idea of cross-validation between different kinds of datasets; Section 3 introduces the triplet loss function, the convolutional neural network model, and evaluation indexes used in this work; Section 4 gives the corresponding results of finger vein verification of training-validation sets, and a brief discussion is given based on the results; finally, the Conclusions of this paper are given.

## 2. Datasets, Preprocessing, and Cross-Validation

### 2.1. Datasets

Three public finger vein datasets employed in this experiment are introduced as follows. *FV-USM database* [13]: the FV-USM database collects finger vein images of 4 fingers of 123 volunteers from Universiti Sains Malaysia. The 4 fingers include the index and middle finger of both hands, and 6 pictures are captured for each finger. There are 492 (123 × 4) classes of fingers and 6 instances for each class. The raw images have the resolution of 640 × 480 pixels. There are extracted ROI (Region of Interest) images (300 × 100 pixels) in the database which are employed directly in this experiment.

*HKPU database* [14]: the HKPU database has 156 subjects and collects 6 finger vein images of the index and middle finger of the left hand for each subject, namely, the database has 312 (156 × 2) classes of fingers and 6 instances for each class. The resolution of the raw images is 513 × 256 pixels.

*SDUMLA-HMT database* [15]: the SDUMLA-HMT database is a multimodal biometric database produced by Shandong University. The finger vein database is part of the SDUMLA-HMT database and consists of finger vein images of 6 fingers of 106 individuals. The 6 fingers include the index, middle, and ring fingers of both hands. There are 6 finger vein images for each finger, namely, the finger vein database has 636 (106 × 6) classes and 6 instances for each class. The resolution of the images of this database is 320 × 240 pixels.  Figure 1 shows the original finger vein samples in the HKPU database and SDUMLA-HMT database. In the images, you can see the tilt of the finger posture and the background noise of the acquisition device. In Table 1, the details of public finger vein datasets employed in this experiment are given in tabular form. It should be noted that the order of resolutions from the highest to the lowest is FV-USM, HKPU, and SDUMLA.

### 2.2. Preprocessing

As described above, there are extracted ROI images in the FV-USM database which are employed directly in this experiment. The HKPU and SDUMLA-HMT databases need to extract ROI images. Because the raw images of the HKPU and SDUMLA-HMT databases are influenced by the edge of the instrument. If we directly detect the edge of the finger using the Sobel operator that can detect edges of a figure by calculating gradients, the edge of the instrument will also be detected. We found that the image of the middle of the finger is almost unaffected by the edge of the instrument, so we use the Sobel operator to detect the edge of the middle of the finger first. Because the edge of the finger is continuous, we gradually extend from the edge of the middle of the finger to the left and right sides to find the edge of the entire finger. We find the middle line of the finger according to the edge of the finger found, and then rotate the finger to the horizontal direction according to the angle between the middle line of the finger and the horizontal direction [4]. Then according to the edge of the finger, the inscribed rectangle is cropped as the ROI of the finger vein. In Figure 2, the preprocessed image samples corresponding to Figure 1 are given. It should be noted that we calculated the mean and standard deviation of each dataset and normalized the images to speed up the convergence of the model.

### 2.3. Cross-Validation

In this experiment, the cross-validation of interdataset is employed in this experiment, and we consider not doing cross-validation of intradataset. Although, the training set and the validation sets of intradatasets are not the same; in fact, the training set and the validation sets of one dataset are from the same input space, and there is no difficult transforming the same input space into feature space by the trained model. The cross-validation of interdataset is employed in the experiment; we use a kind of dataset to train the model, and the other kinds of dataset to validate the model; the input spaces of the training set and the validation sets are different and uncorrelated. We believe that this verification method can better test the recognition ability of the model and is more in line with the actual application scenario of finger vein verification.

## 3. Triplet Loss and Convolutional Neural Networks and Evaluation Indexes

### 3.1. Triplet Loss

The model uses a triplet loss function to learn better feature space representations. The triplet loss function has been explained in detail in the paper [16]; here, we only give a brief description. The calculation of the triplet loss function requires standard or anchor samples, positive samples, and negative samples. The goal of the model training is to make the distance of embedding between positive samples and standard samples smaller than the distance of embedding between negative samples and standard samples, as seen in Figure 3. The kind of positive sample is same as the kind of standard sample, that is, the same finger, and the kind of negative sample is different from the kind of standard sample. The loss function formula is defined as follows

(1) $$\begin{array}{c} L=\overset{N}{\underset{i}{\sum }}{\left[{\left\|f\left(x_{i}^{a}\right)-f\left(x_{i}^{p}\right)\right\|}_{2}^{2}-{\left\|f\left(x_{i}^{a}\right)-f\left(x_{i}^{n}\right)\right\|}_{2}^{2}+\alpha \right]}_{+}. \end{array}$$

*f*(*x*) is the representation of the feature space, *x*_*i*_^*a*^ is the standard sample of the input space, *x*_*i*_^*p*^ is the positive sample of the input space, *x*_*i*_^*n*^ is the negative sample of the input space, and *α* is the interval hyperparameter of the distance between the positive sample and the standard sample and the distance between the negative sample and the standard sample. “+” means that when the value in “” is greater than zero, the value is taken as the loss, and when it is less than zero, the loss is zero. In other words, the triplet we need is the case where the distance of the positive example is greater than the distance of the negative example, and the triplet with the distance of the positive example less than the distance of the negative example is the target of the model training, which is not helpful for the training of the model.

Triplets can be divided into three categories [16], easy triplets are triplets that make loss = 0, i.e., ‖*f*(*x*_*i*_^*a*^) − *f*(*x*_*i*_^*p*^)‖_2_^2^ + *α* < ‖*f*(*x*_*i*_^*a*^) − *f*(*x*_*i*_^*n*^)‖_2_^2^, and such triplets are not helpful for training. Hard triplets are triplets that meet the conditions ‖*f*(*x*_*i*_^*a*^) − *f*(*x*_*i*_^*n*^)‖_2_^2^ < ‖*f*(*x*_*i*_^*a*^) − *f*(*x*_*i*_^*p*^)‖_2_^2^ and must be misidentified, but there are often very few triplets that meet this condition. Semihard triplets, which satisfy the condition ‖*f*(*x*_*i*_^*a*^) − *f*(*x*_*i*_^*p*^)‖_2_^2^ < ‖*f*(*x*_*i*_^*a*^) − *f*(*x*_*i*_^*n*^)‖_2_^2^ < ‖*f*(*x*_*i*_^*a*^) − *f*(*x*_*i*_^*p*^)‖_2_^2^ + *α*, are also the triplets used in the experiments. As shown in Table 2, as the model training progresses, there are fewer and fewer triplets satisfying the semihard condition, which also shows that the model is getting better and better. In Figure 4, the variation of the number of valid training triplets as the training epoch increases is given. It can be found that the number of valid training triplets decreases rapidly in the first few epochs, indicating that the triplet loss function is used as the loss function when training the model; the convergence speed of the model in the first few training epochs is very fast, and as the training epoch increases, the convergence speed gradually slows down.

This experiment adopts the method of generating triplet datasets online [16]. Of course, many of the generated triplet datasets are easy triplets, and not many meet the conditions of semihard triplets. We used the same format as the “pairs.txt” file described in the paper to generate validation sets containing homogeneous and inhomogeneous combinations to verify the performance of the model [17].

### 3.2. Convolutional Neural Networks

In the experiment, a modified 18-layer residual network is trained to represent the transformation from the input space to the feature space, that is, *f*(*x*) in the Equation (1). The detailed structure of ResNet18 has been described in detail in the paper [18–20]. We only give the structure of the weight layer in Table 3. It can be seen that in the last linear transformation layer, the output of the network is the dimension 512 of the feature, not the classification number. Compared with the original ResNet18, the model only transforms the last linear layer from 512 to the embedding of features, instead of the number of categories. The structure of each other layer is identical to that of the original ResNet18. The model is trained to map the input image into the embedding with dimension 512 that can represent the finger vein image well. Determine whether it is the same finger vein by comparing the Euclidean distance of the embeddings with the threshold. If the Euclidean distance between two embeddings is less than the chosen threshold, the two finger veins are the same, and if the Euclidean distance between two embeddings is more than the chosen threshold, the two finger veins are different. This network model is trained with the triplet loss function to get a good representation of the feature space.

The experiment also trains a modified VGGNet16 model [21–23], and the structure of the weight layer of the model is given in Table 4. We added a BatchNorm layer between the convolutional layer and the ReLU (Rectified Linear Unit) activation layer of the original VGGNet16 model. BatchNorm layers can solve the gradient vanishing or explosion problem to a certain extent and speed up the convergence of the model by normalizing the output data. From Table 4, we can see that the modified VGGNet16 model has only one linear transformation layer compared with the original VGGNet16 model which has three linear transformation layers. The original VGGNet16 model, finally, has three layers of linear transformation. The dimensions of features are transformed from maxpool layer 7 × 7 × 512 to 4096, then from 4096 to 4096, and finally from 4096 to the number of classifications. This model only preserves one linear layer to transform the dimensions of features from 7 × 7 × 512 to the uniform feature embedding 512. The structure of each other layer is identical to that of the original VGGNet16. This linear transformation layer is used to transform the extracted feature to embedding of dimension 512. It should be noted that the preprocessing finger vein images are resized to 224 × 224, and the mean and standard deviation of each dataset are calculated to normalize the images. The normalization procedure can speed up the convergence of the model.

### 3.3. Evaluation Indexes

Calculated evaluation indexes used to evaluate the quality of the model are given in Section 4. The definition of these evaluation indexes including accuracy, precision, recall, ROC AUC, and true accept rate would be given as follows. First, the definitions of the four basic indexes are given. TP (true positive), the sample is actually positive and identified as a positive. FN (false negative), the sample is actually positive and identified as a negative. TN (true negative), the sample is actually negative and identified as a negative. FP (false positive), the sample is actually negative and identified as a positive. Accuracy is defined as follows:

(2) $$\begin{array}{c} \text{accuracy}=\frac{\text{TP}+\text{TN}}{\text{TP}+\text{FN}+\text{FP}+\text{TN}}. \end{array}$$

The definition of precision is

(3) $$\begin{array}{c} \text{precision}=\frac{\text{TP}}{\text{TP}+\text{FP}}. \end{array}$$

The definition of recall (also called true positive rate, TPR) is

(4) $$\begin{array}{c} \text{recall}=\frac{\text{TP}}{\text{TP}+\text{FN}}. \end{array}$$

The full name of the ROC curve is the receiver operating characteristic curve. Its vertical axis is TPR, and the horizontal axis is FPR (false positive rate) defined as

(5) $$\begin{array}{c} \text{FPR}=\frac{\text{FP}}{\text{FP}+\text{TN}}. \end{array}$$

The method of drawing the ROC curve is to draw different FPRs and their corresponding TPRs by adjusting the threshold. AUC refers to the area under the ROC curve. By integrating the ROC curve, the AUC can be calculated. The larger the AUC, the better the corresponding performance of the model.

The Euclidean distance of two finger vein images *D*(*x*_*i*_, *x*_*j*_) and the threshold *d* determine the classification of same and different. *N*_same_ is all finger veins pairs (*i*, *j*) of the same finger, and *N*_diff_ is all pairs of different fingers. All true accepts are defined as

(6) $$\begin{array}{c} \text{TA}\left(d\right)=\left\{\left(i,j\right)\in N_{\text{same}},\text{with }D\left(x_{i},x_{j}\right)\leq d\right\}. \end{array}$$

These are the finger pairs (*i*, *j*) that were correctly classified as same at threshold *d*. Similarly

(7) $$\begin{array}{c} \text{FA}\left(d\right)=\left\{\left(i,j\right)\in N_{\text{diff}},\text{with }D\left(x_{i},x_{j}\right)\leq d\right\}, \end{array}$$

is the set of all pairs which was incorrectly classified as same (false accept). The true accept rate TAR(*d*) and the false accept rate FAR(*d*) for a given threshold *d* are defined as [16]

(8) $$\begin{array}{c} \text{TAR}\left(d\right)=\frac{\left|\text{TA}\left(d\right)\right|}{\left|N_{s\text{ame}}\right|},\\ \text{FAR}\left(d\right)=\frac{\left|\text{FA}\left(d\right)\right|}{\left|N_{\text{diff}}\right|}. \end{array}$$

## 4. Results and Discussion

In this experiment, the CNN model training and validation are performed using a Linux server with Intel® Xeon® Gold 5218R CPU @ 2.10GHz (4CPUs), 512GB memory, and NVIDIA GeForce RTX 3090 graphics cards having a memory of 24GB (4GPUs). The experimental models are all implemented under the Pytorch framework, and the models are trained using the backpropagation algorithm and the AdaGrad optimizer [24].

In Tables 5 and 6, the accuracy, precision, recall, ROC AUC (area under the receiver operating characteristic curve), and best distance/threshold of the corresponding training-validation sets are given, respectively, in ResNet18 and VGGNet16 models. The TAR (true accept rate) values are also given at FAR (false accept rate) equals 0.001 of the corresponding training-validation sets in the two CNN models. It can be seen that the verification accuracies of the finger vein are above 92%, the values of precision are all above 94%, the recall values are all above 90%, and the ROC AUC values are above 0.98 in both models, indicating that the trained models have good verification effect and robustness.

We plot the accuracy and ROC AUC of the same training set corresponding to different validation sets in Figure 5; the accuracy and ROC AUC are the average of different validation sets. For example, “F-^∗^” means the training set is FV-USM dataset and the validation sets are the other two datasets; the values are the average of corresponding validation sets, as seen in Figure 5. We can find that for different validation sets, the model obtained from the SDUMLA-HMT training set is better than the model obtained from the HKPU training set, and the model obtained from the HKPU training set is better than the model obtained from the FV-USM training set. The same result can be seen in Figure 5(b). It should be noted that the results of the ResNet18 model in Figures 5(a) and 5(b) are better than the results of the VGGNet16 model, because the residual structure in the ResNet18 model can alleviate the degradation problem in the deep network.

We also plot the accuracy and ROC AUC of the same validation set corresponding to different training sets in Figure 6; accuracy and ROC AUC are the average of different training sets. For example, “^∗^-F” means the validation set is FV-USM dataset and the training sets are the other two datasets; the values are the average of corresponding training sets, as seen in Figure 6. We can find that for different training sets, the results obtained by FV-USM as a validation set are better than those obtained by HKPU as a validation set, and the results obtained by HKPU as a validation set are better than those obtained by SDUMLA-HMT as a validation set. The same result can be seen in Figure 6(b). The results of the ResNet18 model in Figures 6(a) and 6(b) also are better than the results of the VGGNet16 model because of the residual structure in the ResNet18 model.

We found that the trend of the curve in Figures 5 and 6 is just opposite. The curve in Figure 5 shows an upward trend, and the curve in Figure 6 shows a downward trend. A simple explanation is given for this phenomenon. The harder the dataset is used to train the model, namely, the dataset used for the validation set gets the worse results, the better and more robust the trained model will be, as shown in Figure 6 and the opposite trend shown in Figure 5.

Through the analysis of Figures 5 and 6, it can be concluded that SDUMLA-HMT dataset is the most suitable for training set, and FV-USM dataset is the most suitable for testing set. We also notice that the resolution of the SDUMLA-HMT dataset is the lowest, while that of FV-USM dataset is the highest, which illustrates a fact. If the image resolution is lower, the deep learning model will learn more deep features from the image; on the contrary, if the image resolution is higher, the deep learning model will learn fewer deep features from the image. This is consistent with the need to step out of our comfort zone in order to improve ourselves.

The ROC curves of ResNet18 and VGGNet16 models are shown in Figures 7 and 8. It can be seen that the trained models all have ROC AUC values close to 1, i.e., the shape of the ROC curve is close to a square, which also shows that the model can map the input space of the finger vein into the feature space well. It should be noted that in the lower left corner of Figures 7 and 8, the training set is FV-USM, the test set is SDUMLA-HMT, and the ROC curve is the least square, because this situation has the worst training set and testing set.

## 5. Conclusions

- In this experiment, the triplet loss function is applied to the verification of finger veins, and the output embedding of the trained model can represent the features of finger veins well. Good experimental results are obtained, the accuracies of the ResNet18 and VGGNet16 models are at least 92%, and the accuracy of the highest model can even reach 98%, and the ROC AUC values are above 0.98.
- It is worth mentioning that our training set and validation set are completely unrelated, and we use a cross-validation method on different kinds of datasets, so the resulting model is more adaptable. From the results of this experiment, we find that the harder the dataset to identify is used to train the model, the better and more robust the resulting model will be.

## Figures and Tables

**Figure 1:** (a) Finger vein sample from the HKPU database; (b) finger vein sample from the SDUMLA-HMT database.

**Figure 2:** (a) Preprocessed image in the HKPU database; (b) preprocessed image in the SDUMLA-HMT database (corresponding to Figure 1).

**Figure 3:** How the deep learning finger vein verification model computes the finger vein embedding.

**Figure 4:** The variation of the number of valid training triplets as the training epoch increases (an example from this experiment).

**Figure 5:** (a) The accuracy as the same training set in the two CNN models; (b) the ROC AUC value as the same training set in the two CNN models.

**Figure 6:** (a) The accuracy as the same validation set in the two CNN models; (b) the ROC AUC value as the same validation set in the two CNN models.

**Figure 7:** The ROC curve of the corresponding training-validation set in the ResNet18 model.

**Figure 8:** The ROC curve of the corresponding training-validation set in the VGGNet16 model.

**Table 1:** Details of public finger vein datasets employed in this experiment.

Database	Subjects	No. of fingers	Details of fingers	Images per finger	Image size	Total images
FV-USM	123	4	Left & right hand index & middle finger	6	640 × 480	2952
HKPU	156	2	Left hand index & middle finger	6	513 × 256	1872
SDUMLA	106	6	Left & right hand index, middle & ring finger	6	320 × 240	3816

**Table 2:** Number of valid training triplets as the training epoch increases (an example from this experiment).

Epoch	1	2	3	4	5	6	7	8	9	10
No. of valid training triplets	9943	1338	725	502	344	273	256	178	155	151
Epoch	11	12	13	14	15	16	17	18	19	20
No. of valid training triplets	124	122	95	88	76	72	71	70	57	42

**Table 3:** The modified ResNet18 configuration was used in the research.

	Number of filter	Size of feature map	Size of kernel	Number of stride	Number of padding
Image input layer		224(height) × 224(width) × 1(channel)			
Conv1	64	112 × 112 × 64	7 × 7	2 × 2	3 × 3
Maxpool1	1	56 × 56 × 64	3 × 3	2 × 2	1 × 1
Conv2	64	56 × 56 × 64	3 × 3	1 × 1	1 × 1
Conv3	64	56 × 56 × 64	3 × 3	1 × 1	1 × 1
Conv4	64	56 × 56 × 64	3 × 3	1 × 1	1 × 1
Conv5	64	56 × 56 × 64	3 × 3	1 × 1	1 × 1
Conv6	128	28 × 28 × 128	3 × 3	2 × 2	1 × 1
Conv7	128	28 × 28 × 128	3 × 3	1 × 1	1 × 1
Conv8	128	28 × 28 × 128	3 × 3	1 × 1	1 × 1
Conv9	128	28 × 28 × 128	3 × 3	1 × 1	1 × 1
Conv10	256	14 × 14 × 256	3 × 3	2 × 2	1 × 1
Conv11	256	14 × 14 × 256	3 × 3	1 × 1	1 × 1
Conv12	256	14 × 14 × 256	3 × 3	1 × 1	1 × 1
Conv13	256	14 × 14 × 256	3 × 3	1 × 1	1 × 1
Conv14	512	7 × 7 × 512	3 × 3	2 × 2	1 × 1
Conv15	512	7 × 7 × 512	3 × 3	1 × 1	1 × 1
Conv16	512	7 × 7 × 512	3 × 3	1 × 1	1 × 1
Conv17	512	7 × 7 × 512	3 × 3	1 × 1	1 × 1
AdaptiveAvgPool2d		1 × 1 × 512			
Linear (512, 512)		512			

**Table 4:** The modified VGGNet16 configuration was used in the research.

	Number of filter	Size of feature map	Size of kernel	Number of stride	Number of padding
Image input layer		224(height) × 224(width) × 1(channel)			
Conv1	64	224 × 224 × 64	3 × 3	1 × 1	1 × 1
Conv2	64	224 × 224 × 64	3 × 3	1 × 1	1 × 1
Maxpool1	1	112 × 112 × 64	2 × 2	2 × 2	0 × 0
Conv3	128	112 × 112 × 128	3 × 3	1 × 1	1 × 1
Conv4	128	112 × 112 × 128	3 × 3	1 × 1	1 × 1
Maxpool2	1	56 × 56 × 128	2 × 2	2 × 2	0 × 0
Conv5	256	56 × 56 × 256	3 × 3	1 × 1	1 × 1
Conv6	256	56 × 56 × 256	3 × 3	1 × 1	1 × 1
Conv7	256	56 × 56 × 256	3 × 3	1 × 1	1 × 1
Maxpool3	1	28 × 28 × 256	2 × 2	2 × 2	0 × 0
Conv8	512	28 × 28 × 512	3 × 3	1 × 1	1 × 1
Conv9	512	28 × 28 × 512	3 × 3	1 × 1	1 × 1
Conv10	512	28 × 28 × 512	3 × 3	1 × 1	1 × 1
Maxpool4	1	14 × 14 × 512	2 × 2	2 × 2	0 × 0
Conv11	512	14 × 14 × 512	3 × 3	1 × 1	1 × 1
Conv12	512	14 × 14 × 512	3 × 3	1 × 1	1 × 1
conv13	512	14 × 14 × 512	3 × 3	1 × 1	1 × 1
Maxpool5	1	7 × 7 × 512	2 × 2	2 × 2	0 × 0
Linear (25088, 512)		512			

**Table 5:** The accuracy, precision, recall, ROC AUC, and best distance of corresponding training-validation sets in ResNet18 model. The TAR values at FAR = 0.001.

Training-validation	Accuracy	Precision	Recall	ROC AUC	Best distances	TAR
FV-USM-HKPU (F-H)	0.9739 ± 0.0043	0.9762 ± 0.0060	0.9715 ± 0.0084	0.9965	0.6690 ± 0.0030	0.8904
FV-USM-SDUMLA-HMT (F-S)	0.9476 ± 0.0046	0.9563 ± 0.0053	0.9382 ± 0.0049	0.9888	0.5220 ± 0.0060	0.7206
HKPU-FV-USM (H-F)	0.9807 ± 0.0050	0.9890 ± 0.0039	0.9722 ± 0.0072	0.9973	0.5800 ± 0.0000	0.9177
HKPU-SDUMLA-HMT (H-S)	0.9638 ± 0.0035	0.9696 ± 0.0038	0.9575 ± 0.0054	0.9927	0.6100 ± 0.0000	0.8027
SDUMLA-HMT-FV-USM (S-F)	0.9780 ± 0.0052	0.9827 ± 0.0100	0.9734 ± 0.0045	0.9975	0.5700 ± 0.0245	0.8884
SDUMLA-HMT-HKPU (S-H)	0.9713 ± 0.0059	0.9837 ± 0.0094	0.9587 ± 0.0079	0.9958	0.5800 ± 0.0000	0.8503

**Table 6:** The accuracy, precision, recall, ROC AUC, and best distance of corresponding training-validation sets in VGGNet16 model. The TAR values at FAR = 0.001.

Training-validation	Accuracy	Precision	Recall	ROC AUC	Best distances	TAR
FV-USM-HKPU (F-H)	0.9739 ± 0.0068	0.9759 ± 0.0066	0.9718 ± 0.0085	0.9958	0.7700 ± 0.0000	0.8821
FV-USM-SDUMLA-HMT (F-S)	0.9283 ± 0.0063	0.9481 ± 0.0101	0.9063 ± 0.0058	0.9801	0.6290 ± 0.0070	0.6750
HKPU-FV-USM (H-F)	0.9755 ± 0.0052	0.9824 ± 0.0081	0.9685 ± 0.0098	0.9968	0.6190 ± 0.0181	0.9343
HKPU-SDUMLA-HMT (H-S)	0.9462 ± 0.0042	0.9628 ± 0.0153	0.9288 ± 0.0098	0.9879	0.6630 ± 0.0329	0.7478
SDUMLA-HMT-FV-USM (S-F)	0.9723 ± 0.0044	0.9781 ± 0.0068	0.9663 ± 0.0099	0.9953	0.5720 ± 0.0275	0.8896
SDUMLA-HMT-HKPU (S-H)	0.9710 ± 0.0052	0.9861 ± 0.0058	0.9554 ± 0.0094	0.9954	0.6210 ± 0.0070	0.8574

## Data Availability

The experimental datasets are all publicly available online.
